The article "Identification and Validation of a Tumor Microenvironment-Related Gene Signature for Prognostic Prediction in Advanced-Stage Non-Small-Cell Lung Cancer" was published in 2021. Journal: Biomed Res Int.

# Identification and Validation of a Tumor Microenvironment-Related Gene Signature for Prognostic Prediction in Advanced-Stage Non-Small-Cell Lung Cancer

**DOI:** 10.1155/2021/8864436

**Published:** 2021-03-30

**Authors:** Xuening Zhang, Xuezhong Shi, Hao Zhao, Xiaocan Jia, Yongli Yang

**Affiliations:** ^1^Department of Epidemiology and Biostatistics, College of Public Health, Zhengzhou University, Zhengzhou 450001, China; ^2^Zhengzhou University Library, Zhengzhou University, Zhengzhou 450001, China

## Abstract

The development of immunotherapy has greatly changed the advanced-stage non-small-cell lung cancer (NSCLC) treatment landscape. The complexity and heterogeneity of tumor microenvironment (TME) lead to discrepant immunotherapy effects among patients at the same pathologic stages. This study is aimed at exploring potential biomarkers of immunotherapy and accurately predicting the prognosis for advanced NSCLC patients. RNA-seq data and clinical information on stage III/IV NSCLC were obtained from The Cancer Genome Atlas (TCGA) and Gene Expression Omnibus (GEO). In TCGA-NSCLC with stage III/IV (*n* = 192), immune scores and stromal scores were calculated by using the ESTIMATE algorithms. Univariate, LASSO, and multivariate Cox regression analyses were performed to screen prognostic TME-related genes (TMERGs) and constructed a gene signature risk score model. It was validated in external dataset including GSE41271 (*n* = 91) and GSE81089 (*n* = 36). Additionally, a nomogram incorporating TMERG signature risk score and clinical characteristics was established. Further, we accessed the proportion of 22 types of tumor-infiltrating immune cells (TIIC) from the CIBERSORT website and analyzed the difference between two risk groups. OS of patients with high immune/stromal scores were higher (log-rank *P* = 0.044/log-rank *P* = 0.048). Multivariate Cox regression identified six prognostic TMERGs, including CD200, CHI3L2, CNTN1, CTSL, FYB1, and SLC52A1. We developed a six-gene risk score model, which was validated as an independent prognostic factor for OS (HR: 3.32, 95% CI: 2.16-5.09). Time-ROC curves showed useful discrimination for TCGA-NSCLC cohort (1-, 2-, and 3-year AUCs were 0.718, 0.761, and 0.750). The predictive robustness was validated in the external dataset. The C-index and 1-, 2-, and 3-year AUCs of nomogram were the largest, which demonstrated the nomogram had the greatest predictive accuracy and effectiveness and could be used for clinical guidance. Besides, the increased infiltration of T cells regulatory (Tregs) and macrophages M2 in the high-risk group suggested that chronic inflammation may reduce survival probability in patients with advanced NSCLC. We conducted a comprehensive analysis of the tumor microenvironment and identified the TMERG signature, which could predict prognosis accurately and provide a reference for the personalized immunotherapy for advanced NSCLC patients.

## 1. Introduction

Lung cancer remains the leading cause of cancer morbidity and mortality, according to global cancer statistics. In 2018, there were approximately 2.1 million new lung cancer cases and 1.8 million lung cancer deaths, accounting for 11.6% of all new cases and 18.4% of all cancer deaths, respectively, globally [1]. Unfortunately, almost 85% of lung cancer patients are diagnosed with non-small-cell lung cancer (NSCLC) [2]. Among them, 20% of patients belong to stage I/II, and surgical resection is considered as the mainly preferred treatment option. Meanwhile, 80% of patients were diagnosed as stage III/IV, at which time surgery resect no longer available and radiotherapy and chemotherapy are recommended [3]. However, these treatments often lead to drug resistance and relapse in the advanced stage after long-term treatment [4].

In the past decade, immunotherapy has been increasingly prominent in the comprehensive treatment of advanced NSCLC due to its high efficacy and safety [5, 6]. Multiple inhibitory agents, such as programmed death protein-1 (PD-1) and programmed death molecular ligand-1 (PD-L1), have been approved by the FDA for their significant therapeutic effects on advanced NSCLC in the first- and second-line treatment [7]. Results of patient-reported outcomes with durvalumab after chemoradiotherapy in stage III, unresectable non-small-cell lung cancer (PACIFIC trial) has shown a significant increase in progression-free survival with durvalumab in patients at stage III-NSCLC [8]. This suggests that immunotherapy has been extended from patients with distant metastasis (stage IV) to locally advanced patients (stage III). An accurate pathological stage is an important basis for selecting lung cancer treatment. Nevertheless, the complexity and heterogeneity of tumor immunosuppressive microenvironment led to discrepant immunotherapy effects among patients at the same pathologic stages [9]. For particular individuals, the survival benefits of immunotherapy are minimal and with side effects. Therefore, an accurate predictive model is urgently needed to evaluate the prognosis of immunotherapy in patients with advanced NSCLC. Only in this way, appropriate treatments could be selected to balance side effects and survival benefits and to decide whether to implement immunotherapy. No effective biomarkers have been found to independently predict the efficacy of immunotherapy for stage III/IV NSCLC. The development of high throughput technology and bioinformatics makes it possible to find more effective biomarkers in the big data environment.

In the tumor microenvironment, the immune and stromal components together with their secretory factors create a chronic inflammation, immunosuppressive, and tumor-generating environment [10]. The immunotherapy positive response usually depends on the interaction between tumor cells and immune regulation in the tumor microenvironment (TME). Immune and stromal cells are the two main nontumor components of TME [11]. Among these, immune cells are associated with tumor invasion and metastasis, and stromal cells have an important effect on tumor growth, progression, and drug resistance [12, 13]. Our study employed the ESTIMATE algorithm proposed by Yoshihara et al. [14] to calculate the stromal score, immune score, and tumor purity. The algorithm has been used to screen immune- and stromal-related prognostic genes in gastric cancer, liver cancer, and renal cancer, while immune/stromal score in advanced NSCLC based on this algorithm has not been explored [15–17]. Several studies have indicated immune cell infiltration is conducive to explain the pathogenesis and progression of NSCLC. We used the CIBERSORT algorithm proposed by Newman et al. to analyze the immune cell infiltration. The CIBERSORT algorithm could comprehensively, rapidly, and accurately infer the relative proportion of 22 infiltrating immune cells in tissues compared with immunohistochemical technique and flow cytometry [18].

The primary aim of the present study was to identify TME-related genes based on the ESTIMATE algorithm and to construct and validate a TME-related prognostic score model for stage III/IV NSCLC. Secondly, a nomogram which incorporated the TME-related biomarkers and clinical features was constructed to assess the immunotherapy sensitivity and prognostic characteristics for each patient. Finally, we explored the relationship between immune cell infiltration and TME-related risk score model, so as to verify the reliability of the model.

## 2. Materials and Methods

### 2.1. Data Download and Processing

The gene expression data of lung cancer tissues was downloaded from The Cancer Genome Atlas (TCGA) up to July 11, 2020 (https://portal.gdc.cancer.gov/), by using the Genomic Data Commons (GDC, https://portal.gdc.cancer.gov/) tool. The download conditions of the expression profiles for tumors were as follows: (1) primary site was “bronchus and lung”; (2) disease types were “Adenomas and Adenocarcinomas” and “Cystic, Mucinous, and Serous Neoplasms”; (3) projects were “TCGA-LUAD,” “TCGA-LUSC,” and “TCGA-MESO.” Demographic information and clinical pathologic data for the NSCLC patients, including age, gender, race, histology classification, tumor location, tumor stage, T/N/M stage, overall survival (OS) time, overall survival status, progression-free survival (PFS) time, and progression-free survival status, were retrieved and downloaded from the website of cBioPortal (http://www.cbioportal.org/). Based on the requirement to research purpose and data integrality, inclusion criteria were as follows: (1) pathological stages were stage III, stage IIIa, stage IIIb, and stage IV; (2) disease types were lung adenocarcinoma (LUAD), lung squamous cell carcinoma (LUSC), and mesothelioma (MESO). Exclusion criteria are as follows: (1) repeated measurements; (2) missing follow-up time, and tumor stage information; (3) follow-up time was 0 days. Finally, our study identified 192 tumor samples as training dataset. Fragments per kilobase million (FPKM) data were translated into transcripts per million (TPM) data. After deleting duplicate records and expression quantification of TPM data, 19,745 protein-coding genes remained.

Two microarray cohorts, the GSE41271 and the GSE81089 datasets, were selected as external validation. Raw data and annotation files were downloaded from the Gene Expression Omnibus (GEO) (http://www.ncbi.nlm.nih.gov/geo/). Clinical information was retrieved from the website of Sangerbox (http://sangerbox.com/Index). After deleting samples with a follow-up time of 0 and stage I/II, our study finally included 91 and 36 patients from two datasets, respectively. The raw data were processed by RMA background correction, log2 transformation, and normalization by using the “affy” package. Since all data were downloaded from publicly available databases, no ethical approval was required.

### 2.2. Identification of Immune and Stromal-Related DEGs

The ESTIMATE algorithm (https://sourceforge.net/projects/estimateproject/) was used to calculate immune scores, stromal scores, and ESTIMATE scores [14]. We used the “maxstat” statistic to identify the optimal cut-point for continuous variables, which could be achieved through the “survminer” package [19]. Immune and stromal scores were classified into high- and low-score groups according to the optimal cut-off values, respectively. The Kaplan-Meier (K-M) survival curve was used to estimate OS probability, and the log-rank test was employed to compare survival differences between the two groups.

Differential expression analysis of high- and low-score groups was performed with a “limma” package [20]. The *P* value was adjusted by the false discovery rate (FDR) [21]. The up- and downregulated genes of immune and stromal were obtained based on the criteria of fold change ≥ 1.5 and adjusted FDR < 0.05. The intersection between immune-related differentially expressed genes (DEGs) and stromal-related DEGs was identified by using the VENNY online website (https://bioinfogp.cnb.csic.es/tools/venny/). Heat maps and volcano plots of DEGs were realized by the “pheatmap” package and “ggplot2” package.

### 2.3. Function and Pathway Enrichment Analysis of DEGs

The Gene Ontology (GO) and Kyoto Encyclopedia of Genes and Genomes (KEGG) pathway enrichment analysis of DEGs could be implemented by the Database for Annotation, Visualization and Integrated Discovery (DAVID, https://david-d.ncifcrf.gov/) [22–24]. GO analysis included three main parts of biological process (BP), cellular component (CC), and molecular function (MF). We selected the top ten of GO terms in three parts to draw the histogram. The top fifteen KEGG analysis terms were exhibited in the bubble chart (adjusted *P* value < 0.05 was statistically significant).

### 2.4. Construction and Validation of the TMERG Prognostic Risk Score Model

Firstly, a univariate analysis of differential genes was performed to screen out significant genes. Subsequently, the least absolute shrinkage and selection operator (LASSO) Cox regression model was utilized for the further screen prognostic genes to reduce redundant genes and avoid overfitting the model. Finally, a Cox stepwise regression analysis was served to determine all independent prognostic genes in the model [25]. The formula of TMERG signature is as follows: risk score = *∑* (*βi*∗Exp*i*) (*i* represented the rank of prognostic genes, *βi* represented every gene coefficient, and Exp*i* represented every gene expression). Advanced NSCLC were separated into high-risk and low-risk groups according to the optimal cut-point of risk score. The Kaplan-Meier (K-M) survival curve was used to estimate OS probability and PFS probability, and the log-rank test was employed to compare survival time differences between the two groups. “Survival” package, “glmnet” package, “survminer” package, and “forestplot” package were used to conduct the above analysis.

The TMERG signature risk score model was validated by 91 and 36 advanced NSCLC patients from the GSE81089 and GSE41271 datasets. According to the risk score formula of the training set, two independent validation sets were also divided into a high-risk group and a low-risk group, respectively. Similarly, the K-M survival curve and log-rank test were employed to compare survival probability differences between the two groups. The performance of the risk score model in the training set and validation set was assessed based on the time-dependent ROC, which was realized by “timeROC.” The area under the curve (AUC) is more than 0.6, indicating good prediction discrimination.

### 2.5. Construction of Nomogram and Performance Assessment

In order to assess the independent prognostic effect of TMERG signature, all possible prognostic factors, including demographic, clinical-pathological characteristics, and gene risk score model, were incorporated into univariate and multivariate Cox proportional hazard regression. The results were visualized using the “forestplot” package in R software.

The nomogram could accurately predict the survival probability of an individual patient based on clinical characteristics and TMERG signature risk score and has been widely used in clinical diagnosis and prediction [26]. In the present study, a nomogram was constructed including all meaningful prognostic factors. For each individual, a total score could be calculated by adding up the score of each prognosis factors, thereby predicting 1-, 2-, and 3-year survival probabilities. Subsequently, time-dependent ROC and calibration were used to assess the performance of nomogram, which was realized by the “timeROC” and “rms” package [27]. If probabilities approach the 45-degree angle line in a calibration plot, it indicates that there was a good consistence between the risk score prediction and the actual observations.

### 2.6. Estimated Infiltrating Immune Distribution Based on TMERG Signature

CIBERSORT is a deconvolution algorithm for immune cell subtype expression based on linear support vector regression [18]. LM22 provides the annotated gene expression signatures for 22 immune cell subtypes, including seven T cell types, naive and memory B cells, plasma cells, natural killer (NK) cells, and myeloid subsets. The standardized gene expression data was uploaded to the CIBERSORT website (http://cibersort.stanford.edu/), and the algorithm was run based on LM22 signatures and 1000 arrangements. *P* < 0.05 for the type of immune cells, indicating that the hypothesis of the type of immune cells is accurate, it is considered qualified for further analysis. We evaluated the fractions of tumor immune infiltrating cell (TIIC) type components in every NSCLC sample by using the CIBERSORT algorithm. Unsupervised hierarchical clustering analysis was performed to visualize the proportions of TIIC in high-risk group tissues and low-risk group tissues. The Wilcoxon test was performed to compare the differences of TIIC between high-risk group tissues and low-risk group tissues.

### 2.7. Statistical Analysis

If the sample satisfies normal distribution, an independence *t* test was used to determine the significance of the differences in mean values between the two groups, and a one-way ANOVA test was used for variables in more than two groups. If the sample did not satisfy normal distribution, Wilcoxon is used to compare the two groups of variables, and Kruskal-Wallis was used to compare more than two groups of variables. The K-M survival curve was drawn to calculate survival probability, and the log-rank test was used to determine the significance of the difference in survival probability between the two groups. Correlation coefficient was calculated using Spearman's correlation analyses. All statistical analyses were implemented by R software 3.6.3. *P* < 0.05 was considered as statistically significant.

## 3. Results

### 3.1. Patient Demographic and Clinical Characteristic

The entire training cohort involved gene expression data and clinical information of 192 advanced NSCLC patients from TCGA database. GSE41271 (*n* = 91) and GSE81089 (*n* = 36) were used as two independent verification cohorts. The detailed demographic and clinical pathologic characteristics of the three independent cohorts are listed in Table 1.

### 3.2. Association of Immune and Stromal Scores with Clinical Stage and Prognosis

The ESTIMATE algorithm was applied to estimate the immune scores and stromal scores. Immune scores range from -1181.63 to 3348.10, and stromal scores range from -1805.27 to 1923.43. Both immune and stromal scores roughly increased with increasing tumor invasion stage. Tumors with low invasion (T1) yielded significantly higher stromal and immune scores than those high invasion groups (T2 and T3) (*P* < 0.05). There was no significant difference in immune and stromal scores in different M stages, N stages, and pathological stages (Figure S2).

The optimal cut-off values were calculated by the R package “maxstat.” Advanced NSCLC patients were separated into a high-score group and a low-score group by the optimal cut-off value (Figure S3). According to the log-rank test results, the mean OS time of patients with a high immune score was significantly longer than that of patients with a low immune score (log-rank test *P* = 0.044) (Figure 1(a)). Similarly, patients with a high stromal score had better OS probability than those with a low stromal score (log-rank test *P* = 0.043) (Figure 1(b)). The PFS of the high immune score group was significantly higher than that of the low immune score group (log-rank test *P* = 0.004) (Figure 1(d)). There was no significant difference in PFS between high and low stromal score groups (log-rank test *P* = 0.076) (Figure 1(e)).

### 3.3. Identification of Immune and Stromal-Related DEGs

We used the “limma” package to analyze RNA-expression data. Immune- (or stromal-) related differentially expressed genes (DEGs) were identified by comparing the RNA-expression comparison of NSCLC patients with high and low immune/stromal scores. A cluster analysis screened out immune-related DEGs with high scores and low groups displayed in a heat map (Figure 2(a)). A volcano plot exhibited significantly differentially expressed genes (Figure 2(c)). A total of 1126 immune-related differential genes were identified, which contain 139 upregulated genes and 987 downregulated genes. The heat map and volcano map of stromal-related DEGs are shown in Figures 2(b) and 2(d). A total of 1497 stromal-related DEGs including 302 upregulated genes and 1195 downregulated genes were screened. A Venn diagram displayed 711 intersecting DEGs related to immune and stromal, namely, TME-related DEGs, including 67 upregulated and 644 downregulated genes (Figure 2(e)).

Top terms of GO analysis included immune response, defense response, response to wounding, and inflammatory response in BP; plasma membrane, plasma membrane part, and extracellular region in CC; and carbohydrate binding, cytokine activity, and polysaccharide binding in MF (Figure 2(f)). The results of KEGG enrichment were also related to immune responses, including cytokine-cytokine receptor interaction, chemokine signaling pathway, and cell adhesion molecules (CAMs) (Figure 2(g)). Collectively, these results indicated that the enriched GO terms and KEGG pathways were mainly related to immune response.

### 3.4. Screening of Prognostic TMERG and Construction of TMERG Signature

A total of 77 genes related to the prognosis of advanced NSCLC from 711 DEGs were screened by univariate Cox analysis. LASSO regression analysis models further identified 19 genes associated with OS (Figures 3(a) and 3(b)). Six significant independent prognostic genes were selected by multivariate Cox regression analysis (Figure 3(c)). Among them, CD200, CHI3L2, FYB1, and SLC52A1 were protective genes, whereas CNTN1 and CTSL were risk genes. Patients with high expression of protective four genes have a high survival probability, whereas high expression of two risk genes is associated with lower survival probability (Figure S3). The prognostic gene risk score model = (−0.326 × expression value of CD200) + (−0.187 × expression value of CHI3L2) + (0.111 × expression value of CNTN1) + (0.505 × expression value of CTSL) + (−0.310 × expression value of FYB1) + (−0.252 × expression value of SLC52A1). According to the optimum cut-off threshold of 0.463, all advanced NSCLC patients were separated into a high-risk group (*n* = 68) and a low-risk group (*n* = 124). The differences of OS and PFS in the two risk score groups are significant by the log-rank test (OS: *P* < 0.001; PFS: *P* < 0.001, Figures 3(d) and 3(e)).

According to time-dependent ROC analysis, the AUCs of the OS predicted value in 1-, 2-, and 3-year were 0.718, 0.761, and 0.681. And the AUCs of 1-, 2-, and 3-year were 0.801, 0.827, and 0.784 for the PFS prediction. The results showed that the discrimination of the prognostic model was good.

### 3.5. Validation of TMERG Signature in External Dataset

To verify the predictive robustness of the TMERG signature, its performance was evaluated in two independent external cohorts (GSE41271 and GSE81089). The risk score of each patient in the testing sets was calculated according to the relative expression levels of the six genes, using the same formula established in the training set. In each dataset, samples were divided into a low-risk group and a high-risk group with the optimal cut-off. The OS of patients in the low-risk group was significantly lower than that in the high-risk group (GSE41271: *P* < 0.045; GSE81089: *P* < 0.021, Figures 4(a) and 4(b)).

The evaluation of the validation cohort is based on time-dependent ROC. Results of time-dependent ROC indicated that the AUCs for 1, 2, and 3 years were 0.702, 0.620, and 0.637 in GSE41271 (Figure 4(c)). The AUC values of the six-gene signature in predicting 1-, 2-, and 3-year survival of advanced NSCLC patients were 0.770, 0.641, and 0.680 in GSE81089 (Figure 4(d)). In summary, the prognostic risk score model of advanced NSCLC was verified to be effective and robust.

### 3.6. Construction of Nomogram and Performance Assessment

To determine whether TMERG signature is an independent prognostic factor for patients with advanced NSCLC, TMERGs along with covariates including age, gender, histological type, M stage, N stage, T stage and tumor stage, and smoking history were involved in the univariate and multivariate Cox regression models. The results of univariate and multivariate Cox regression analyses demonstrated that the pathological N stage, pathological T stage, and risk score were independent prognostic factors for advanced NSCLC patients (Figures 5(a) and 5(b)). We constructed a nomogram, combining these independent prognostic factors, as a quantitative approach for calculating survival. Every patient could obtain a total score by adding a corresponding score for each prognostic factor (Figure 6(a)). Higher total scores corresponded to a worse survival probability of patients. Furthermore, the AUCs of the nomogram were 0.720, 0.799, and 0.772 at 1, 2, and 3 years, respectively (Figure 6(b)). Calibration showed that the 1-, 2-, and 3-year probabilities approach the 45-degree angle line, implying that there was a good consistence between the nomogram prediction and the actual observations (Figure 6(c)).

We compared the predictive performance of the nomogram, N stage, T stage, and TMERG risk score model. The result showed the AUCs for nomogram predicting 1-, 2-, and 3-year OS were the largest in all models. The C-index of pathologic N stage, pathologic T stage, risk score model, and nomogram was 0.558, 0.569, 0.639, and 0.703, respectively (Table 2). Taking together, combining our risk score model might increase the predicting sensitivity and specificity of the conventional TNM stage and bring some net benefit, which might help clinical management.

### 3.7. Infiltrating Immune Cell Distribution in Advanced NSCLC

To further confirm the correlation between our TMERG signature and immune microenvironment, we applied the CIBERSORT algorithm to calculate TIIC proportions and construct 22 kinds of TIIC profiles for patients with advanced NSCLC (Figure 7(a)). The difference of the proportion of immune infiltrating cells between high-risk and low-risk samples was displayed in the heat map (Figure 7(b)). The results from the Wilcoxon test showed that a total of four kinds of TIICs were different in two risk score groups (Figure 6(c)). Among them, the immune cells with significantly higher infiltrated in high-risk samples compared with low-risk samples were T cells regulatory (Tregs) and macrophages M2 (*P* < 0.05). T cells CD8 and macrophages M1 were significantly higher in low-risk samples than those in high-risk samples (*P* < 0.05). Therefore, different immune infiltrates in advanced NSCLC patients might be used as prognostic indicators and targets of immunotherapy.

## 4. Discussion

There has been growing awareness in cancer research that cancer is a complex ecosystem composed of both tumor cells and nontumor cells. Nontumor components in tumor tissues form TME. TME can not only promote tumor cell proliferation and protect tumor cells from apoptosis and metastasis but also play a crucial role in immunotherapy. Our study calculated immune scores/stromal scores in TME by using the ESTIMATE algorithm, resulting in immune scores were positively correlated with OS time. The TMERG risk score model involving 6 genes (CD200, CHI3L2, CNTN1, CTSL, FYB1, and SLC52A1) was constructed and validated. Compared with the TNM staging system and single TME-related biomarkers, the multigene comprehensive model has the advantages of accurate prediction and abundant information. The nomogram, combining molecular level and clinical characteristics, may provide more precise prognostic predictions for individuals.

In the present study, we comprehensively elucidated the TME, especially the two nontumor components, namely, immune cells and stromal cells. Immune and stromal scores calculated by the ESTIMATE algorithm clarified the diversity of immune and stromal components in the TME. Our results illustrated that immune and stromal scores were positively correlated with tumor invasion and negatively correlated with survival time in advanced NSCLC patients. This demonstrated from different perspectives that immune/stromal cells within TME play an indispensable role in tumorigenesis.

Immune-related genes and stromal-related genes were overlapped to obtain TME-related genes, which were identified as candidate genes predicting the prognosis of advanced NSCLC and representing the TME pattern. GO analysis shows that 711 TMERGs are involved in immune-related biological processes such as immune response, defense response, response to wounding, and inflammatory response. KEGG analysis revealed DEG enrichment in immune-related pathways including cytokine-cytokine receptor interaction, chemokine signaling pathway, and cell adhesion molecules (CAMs). Functional annotation again demonstrated that the immune- and stromal-related DEGs could be representative of TME patterns and were significantly associated with immune infiltration status in NSCLC.

Univariate, LASSO, and multivariate Cox regression analyses were used to screen the independent prognosis genes to establish a TMERG signature, which had a high accuracy in predicting OS and PFS of advanced NSCLC patients. We found that TCGA-NSCLC patients in the low-risk group had a significantly longer OS and PFS than patients in the high-risk group, and these findings were validated in two independent GEO datasets subsequently. Time-dependent ROC curves and C-index also indicated that the TMERG risk score had a beneficial effect on prognosis prediction. Although AUCs and C-index of the TMERG risk score model were higher than the traditional pathological N and T stage, the nomogram combining the TMERG risk score model and the pathological stage had the best accuracy and resolution.

The six genes that composed the risk score could be considered as potential therapeutic targets. Among these, CD200, CHI3L2, FYB1, and SLC52A1 are the protective factors in the model. CD200 molecule (CD200) is a member of the immunoglobulin superfamily, which is expressed by various cell types, including B cells, T cells, thymocytes, endothelial cells, and neurons [28]. CD200 has been reported to inhibit antitumor responses by modulating the function of macrophages and T cells [29–31]. On the contrary, Yoshimura et al. corroborated that high expression of CD200 is a protective factor for the prognosis of NSCLC [32]. Specifically, the mRNA expression levels of several inflammatory chemokines were significantly increased when CD200 was deleted realized by RT-qPCR. These opposite results suggest that the effect of CD200 depends on the tumor stage and type. Chitinase 3-like protein 2 (CHI3L2), a glycosyl hydrolase family member, encodes a protein similar to bacterial chitinase but lacking chitinase activity. Upregulation of CHI3L2 could increase the phosphorylation level of ERK1 and ERK2, thus inhibiting tumor cell mitosis and proliferation in glial cell tumors [33, 34]. FYN Binding Protein 1 (FYB1) also is known as adhesion and degranulation-promoting adapter protein (ADAP). ADAP is necessary for T cell activation [35]. Recent studies have shown that T cells use ADAP to increase activation and adhesion of *β*2 integrin in cells stimulated by infection or chemokines. In addition, ADAP promotes antitumor response through expression in primary NK cells and il-2-stimulated lymphocyte-activated killer cells [35]. The alias of Solute Carrier Family 52 Member 1 (SLC52A1) is protease-activated receptor 2 (PAR2). PAR2 is a member of G-protein-coupled receptors. PAR2 deletion could reconstruct TME, establish immunosuppressive microenvironment, and promote tumor progression through accumulating protumor medullary cells which include macrophages and marrow-derived suppressive cells and reducing antitumor T cells. The specific mechanism is that PAR2 deficiency directly enhances immunosuppressive activity by promoting production of reactive oxygen species mediated by STAT3 [36]. These studies suggest that PAR2 is a favorable prognostic factor for some cancer.

CNTN-1 and CTSL are independent prognostic risk factors. Contactin-1 (CNTN-1) is a nerve cell adhesion molecule that has been proved to be involved in the development of the nervous system [37]. In recent years, it has been reported that the abnormal expression of CNTN-1 is closely related to the tumor occurrence and progression [38–42]. For example, Chen et al. found that increased expression of CNTN-1 could promote the metastasis of gastric cancer cells [43]. Zhang et al. demonstrated that silencing CNTN-1 could improve the sensitivity of chemotherapy drugs and inhibit the metastasis and invasion of NSCLC tumor cells [44]. Cathepsin L (CTSL), a lysosomal cysteine protease member, is mainly involved in the terminal degradation of intracellular phosphorylated proteins [45]. Increasing evidences indicate that CTSL is highly specifically expressed in various cancers [46–49]. Sullivan et al. found that CTSL promotes tumor cell replication and metastasis by activating epithelial to mesenchymal transition (EMT) gene transcription [46]. Previous studies have also found that inhibition of CTSL could inhibit EMT-mediated invasion and metastasis of NSCLC cells.

Immune cells in TME play key roles in either tumor-promoting or tumor-suppressive effects. Although T cell subsets play an important role in tumor inhibition, some T cell types promote tumor progression through different growth factors [50]. For example, the presence of CD8^+^ and CD4^+^ T cells could improve clinical outcomes and prolong survival in different cancers [51–54], while T cell regulation (Tregs) may inhibit antitumor immune response and support the establishment of immune hyporesponse microenvironments in some tumor types [55]. Macrophages, an important component of TIICs, serve as the key mediator between inflammation and cancer [56, 57]. Macrophages could be differentiated into classical macrophage M1 and substitute macrophage M2, which have antitumor and protumor effects, respectively [58]. According to our results, the Tregs and macrophages M2 accounted for significantly higher proportions in high-risk samples than that in low-risk samples, whereas T cells CD8 and macrophages M1 accounted for significantly higher in low-risk samples than those in high-risk samples. Therefore, we inferred that the upregulated Tregs and macrophages M2 in the high-risk group may contribute to worse prognosis of NSCLC. The low-risk group had a better OS, which may be attributed to the upregulation of CD8^+^ T cells and macrophage M1. To sum up, exploring the regulatory mechanisms of different immune cell types is vital for finding new therapeutic strategies and improving the immunotherapy response of NSCLC.

Nowadays, some studies have been aimed at finding prognostic prediction of patients with advanced non-small-cell lung cancer. He et al. considered that the imaging biomarkers extracted by tumor mutational burden could effectively predict the therapeutic effect of immune checkpoint inhibitors in advanced NSCLC patients [59]. Moik et al. demonstrated that inflammation and hemostasis could serve as biomarkers for unfavorable prognosis and poor therapy response in advanced lung cancer patients [60]. Perrone et al. found that hypercholesterolemia implies a low-grade inflammatory state that could distinguish the best beneficiaries of immunotherapy in NSCLC [61]. Mildner et al. proposed that PD-1^+^ CD4^+^ T cell count and PD-1^+^ CD8^+^ T cells could act as the liquid biomarkers of immunological factors [62]. The present study differed from previous reports about advanced NSCLC prognosis and had its own advantages. Firstly, no study provided a reliable TME-related signature for advanced-NSCLC prognosis. Immunotherapy is the optimal treatment for advanced NSCLC, and the detection of some liquid immune biomarkers is often unstable or impractical, thereby TME-related signature based on the ESTIMATE algorithm may be more comprehensive and effective than other single biomarkers. Secondly, we further demonstrate the diagnostic efficacy of our TME-related signature in two independent external GEO datasets and verify the robustness of the model. Finally, the multivariate Cox regression model adjusted for other clinical covariates, which could demonstrate that TME-related gene signature was an independent prognostic factor for advanced NSCLC patients.

Nevertheless, our current research remains a few limitations. Firstly, the main source of clinical characteristics for our dataset was TCGA database. The majority of patients were from North America, and thus, extending our findings to other races of patients should be with great caution. Secondly, our study provides the evidence that six novel TME-related genes are significantly related to the prognosis of advanced NSCLC patients, which was analyzed through data mining merely. The function and mechanism of these genes depend on further experimental studies to elucidate. In addition, our retrospective study could lead to reporting bias; thus, the result of new TMERG signature needs to be further validated in prospective studies.

## 5. Conclusions

In summary, we have demonstrated the effectiveness of the ESTIMATE algorithm applied to screen TMERG in advanced NSCLC. The single gene of CD200, CHI3L2, CNTN1, CTSL, FYB1, and SLC52A1 and the combination model have been confirmed to have an association with the prognosis of advanced NSCLC patients, and the stability and independence have been verified. We also found that the risk score was related to the immune cell infiltration component, which further authenticated the reliability of the risk score model. The potential interaction among six genes and their predictive value in immunotherapy needs to be validated in prospective cohorts for advanced NSCLC patients.

## Figures and Tables

**Figure 1:** Association of stromal and immune scores with the prognosis of advanced NSCLC in TCGA. Kaplan-Meier survival curves and log-rank test between high and low (a) immune score groups, (b) stromal score groups, and (c) ESTIMATE score groups.

**Figure 2:** Comparison of gene expression profiles between immune and stromal scores in TCGA. (a, b) Heat maps showing expression profiles for immune score and stromal score-related DEGs. (c, d) Volcano plots showing upregulated and downregulated genes for immune score and stromal score related. (e) Venn diagram showing the intersection of the immune score and stromal score-related upregulated/downregulated DEGs. (f) Histogram showing top ten of Gene Ontology terms in BP, CC, and MF. (g) Bubble chart exhibiting top fifteen of KEGG analysis terms.

**Figure 3:** Identification of TME-related genes associated with advanced NSCLC prognosis. (a, b) Seventy-seven TMERGs were identified by a LASSO regression analysis. (c) Forest map showing six independent prognostic genes identified by a multivariate Cox regression analysis. (d, e) Kaplan-Meier survival curves and log-rank test of OS and PFS between high- and low-risk score groups in TCGA. (d, e) The AUC for 1-, 2-, and 3-year predicted OS and PFS in TCGA.

**Figure 4:** Prognostic analysis and performance assessment of GEO external dataset. (a) Kaplan-Meier survival curves and log-rank test of high- and low-risk score groups in GSE41271. (b) Kaplan-Meier survival curves of high- and low-risk score groups in GSE81089. (c) The AUC for 1-, 2-, and 3-year overall survival in GSE41271. (d) The AUC for 1-, 2-, and 3-year predicted OS in GSE81089.

**Figure 5:** Univariate and multivariate Cox regression analysis of prognostic factors in TCGA. (a) Univariate Cox regression analysis of all potential prognostic factors in TCGA. (b) Multivariate Cox regression analysis of all independent prognostic factors in TCGA.

**Figure 6:** Nomogram and performance assessment. (a) Nomogram based on clinical factors and TMERG risk score. (b) The AUC for 1-, 2-, and 3-year predicted OS in nomogram. (c) Calibration for the possibility of 1-, 2-, and 3-year predicted OS in nomogram.

**Figure 7:** Immune infiltrations of high- and low-risk groups in TCGA. (a) Relative proportion of immune infiltration in high- and low-risk groups. (b) Heat map of 22 immune cell proportions in high- and low-risk score groups. (c) Correlation of significantly different immune cells between high- and low-risk score groups.

**Table 1:** The clinical characteristics of advanced NSCLC in training and validation cohort (*n* (%)).

Characteristics	Training set	Validation set	
	TCGA (*n* = 192)	GSE41271 (*n* = 91)	GSE81089 (*n* = 36)
Age (year)			
<65	82 (42.71)	33 (36.26)	13 (36.11)
≥65	110 (57.29)	58 (63.74)	23 (63.89)
Gender			
Male	117 (60.94)	54 (59.34)	14 (38.89)
Female	75 (39.06)	37 (40.66)	22 (61.11)
Histological type			
LUAD	104 (54.17)	55 (60.44)	27 (75)
LUSC	88 (45.83)	36 (39.56)	9 (25)
Metastasis (M_stage)			
M0	160 (83.33)	85 (93.41)	33 (91.67)
M1	32 (16.67)	6 (6.59)	3 (8.33)
Lymph node (N_stage)			
N0	30 (15.63)	—	—
N1	47 (24.48)	—	—
N2	106 (55.21)	—	—
N3	9 (4.69)	—	—
Tumor invasion (T_stage)			
T1	21 (10.94)	—	—
T2	85 (44.27)	—	—
T3	45 (23.44)	—	—
T4	41 (21.35)	—	—
Tumor stage			
III	160 (83.33)	85 (93.41)	33 (91.67)
IV	32 (16.67)	6 (6.59)	3 (8.33)
Smoking			
Yes	166 (86.46)	80 (87.91)	—
No	26 (13.54)	11 (12.09)	—

Abbreviations: LUAD = lung adenocarcinoma; LUSC = lung squamous cell carcinoma.

**Table 2:** Comparison of the nomogram with the N stage, T stage, and risk score model.

Models	1-year AUC (95% CI)	2-year AUC (95% CI)	3-year AUC (95% CI)	C-index (95% CI)
N stage model	0.560 (0.465-0.655)	0.612 (0.532-0.693)	0.566 (0.475-0.657)	0.558 (0.499-0.617)
T stage model	0.576 (0.482-0.669)	0.587 (0.499-0.675)	0.595 (0.496-0.694)	0.569 (0.510-0.628)
Risk score model	0.718 (0.641-0.796)	0.761 (0.695-0.827)	0.750 (0.681-0.818)	0.639 (0.586-0.692)
Nomogram	0.720 (0.629-0.812)	0.799 (0.726-0.872)	0.772 (0.693-0.851)	0.703 (0.650-0.756)

Abbreviations: 95% CI = confidence interval.

## Data Availability

The Cancer Genome Atlas (TCGA) database (https://cancergenome.nih.gov/) is used to provide RNA-seq data and the clinical data of NSCLC in training set . The Gene Expression Omnibus (GEO) (http://www.ncbi.nlm.nih.gov/geo/) is used to provide RNA-seq data in validation set.

## Supplementary Materials

Supplementary 1 Figure S1: association of stromal and immune scores with clinical characteristics advanced NSCLC in TCGA.

Supplementary 2 Figure S2: the optimal cut-off identification for the immune score, stromal score, and ESTIMATE score.

Supplementary 3 Figure S3: Kaplan-Meier survival curves and log-rank test of six prognosis TME-related genes in TCGA.

## References

[1] Bray F., Ferlay J., Soerjomataram I., Siegel R. L., Torre L. A., Jemal A. (2018). Global cancer statistics 2018: GLOBOCAN estimates of incidence and mortality worldwide for 36 cancers in 185 countries. *CA: a Cancer Journal for Clinicians*.

[2] Molina J. R., Yang P., Cassivi S. D., Schild S. E., Adjei A. A. (2008). Non-small cell lung cancer: epidemiology, risk factors, treatment, and survivorship. *Mayo Clinic Proceedings*.

[3] Filippi A. R., Di Muzio J., Badellino S., Mantovani C., Ricardi U. (2018). Locally-advanced non-small cell lung cancer: shall immunotherapy be a new chance?. *Journal of Thoracic Disease*.

[4] Chen Y. T., Feng B., Chen L. B. (2012). Update of research on drug resistance in small cell lung cancer chemotherapy. *Asian Pacific Journal of Cancer Prevention*.

[5] Levy A., Doyen J., Botticella A. (2020). Role of immunotherapy in locally advanced non-small cell lung cancer. *Cancer Radiothérapie*.

[6] Inoue H., Okamoto I. (2019). Immune checkpoint inhibitors for the treatment of unresectable stage III non–small cell lung cancer: emerging mechanisms and perspectives. *Lung Cancer*.

[7] Ancevski Hunter K., Socinski M. A., Villaruz L. C. (2018). PD-L1 testing in guiding patient selection for PD-1/PD-L1 inhibitor therapy in lung cancer. *Molecular Diagnosis & Therapy*.

[8] Antonia S. J., Villegas A., Daniel D. (2017). Durvalumab after chemoradiotherapy in stage III non-small-cell lung cancer. *The New England Journal of Medicine*.

[9] Kim S., Kim A., Shin J. Y., Seo J. S. (2020). The tumor immune microenvironmental analysis of 2,033 transcriptomes across 7 cancer types. *Scientific Reports*.

[10] Gajewski T. F., Schreiber H., Fu Y. X. (2013). Innate and adaptive immune cells in the tumor microenvironment. *Nature Immunology*.

[11] Fridman W. H., Pagès F., Sautès-Fridman C., Galon J. (2012). The immune contexture in human tumours: impact on clinical outcome. *Nature Reviews. Cancer*.

[12] Zhang L., Conejo-Garcia J. R., Katsaros D. (2003). Intratumoral T cells, recurrence, and survival in epithelial ovarian. *The New England Journal of Medicine*.

[13] Straussman R., Morikawa T., Shee K. (2012). Tumour micro-environment elicits innate resistance to RAF inhibitors through HGF secretion. *Nature*.

[14] Yoshihara K., Shahmoradgoli M., Martínez E. (2013). Inferring tumour purity and stromal and immune cell admixture from expression data. *Nature communications*.

[15] Wang H., Wu X., Chen Y. (2019). Stromal-immune score-based gene signature: a prognosis stratification tool in gastric cancer. *Frontiers in oncology*.

[16] Peng-lei Ge S.-f L., Wang W.-w., Li C.-b., Yu-bin F., Feng Z.-k. (2020). Prognostic values of immune scores and immune microenvironmentrelated genes for hepatocellular carcinoma. *Aging (Albany NY)*.

[17] Chen B., Chen W., Jin J., Wang X., Cao Y., He Y. (2019). Data mining of prognostic microenvironment-related genes in clear cell renal cell carcinoma: a study with TCGA database. *Disease Markers*.

[18] Newman A. M., Liu C. L., Green M. R. (2015). Robust enumeration of cell subsets from tissue expression profiles. *Nature Methods*.

[19] Torsten Hothorn A. Z. (2007). Generalized maximally selected statistics. *Biometrics*.

[20] Ritchie M. E., Phipson B. (2015). limma powers differential expression analyses for RNA-sequencing and microarray studies. *Nucleic Acids Research*.

[21] Anat Reiner D. Y., Benjamini Y. (2003). Identifying differentially expressed genes using false discovery rate controlling procedures. *Bioinformatics*.

[22] Ashburner M., Ball C. A., Blake J. A. (2000). Gene Ontology: tool for the unification of biology. *Nature Genetics*.

[23] Kanehisa M., Furumichi M., Tanabe M., Sato Y., Morishima K. (2017). KEGG: new perspectives on genomes, pathways, diseases and drugs. *Nucleic Acids Research*.

[24] Glynn Dennis Jr B. T. S., Hosack D. A., Yang J., Gao W., Lane H. C., Lempicki R. A. (2003). DAVID: Database for Annotation, Visualization, and Integrated Discovery. *Genome Biology*.

[25] Motakis E., Ivshina A. V., Kuznetsov V. A. (2009). Data-driven approach to predict survival of cancer patients: estimation of microarray genes’ prediction significance by Cox proportional hazard regression model. *IEEE Engineering in Medicine and Biology Magazine*.

[26] Iasonos A., Schrag D., Raj G. V., Panageas K. S. (2008). How to build and interpret a nomogram for cancer prognosis. *Journal of Clinical Oncology*.

[27] Alba A. C., Agoritsas T., Walsh M. (2017). Discrimination and calibration of clinical prediction models: users’ guides to the medical literature. *JAMA*.

[28] Barclay A. N., Wright G. J., Brooke G., Brown M. H. (2002). CD200 and membrane protein interactions in the control of myeloid cells. *Trends in Immunology*.

[29] Coles S. J., Wang E. C., Man S. (2011). CD200 expression suppresses natural killer cell function and directly inhibits patient anti-tumor response in acute myeloid leukemia. *Leukemia*.

[30] Wang L., Liu J. Q., Talebian F. (2010). Tumor expression of CD200 inhibits IL-10 production by tumor-associated myeloid cells and prevents tumor immune evasion of CTL therapy. *European Journal of Immunology*.

[31] Zhang S., Cherwinski H., Sedgwick J. D., Phillips J. H. (2004). Molecular mechanisms of CD200 inhibition of mast cell activation. *Journal of Immunology*.

[32] Yoshimura K., Suzuki Y., Inoue Y. (2020). CD200 and CD200R1 are differentially expressed and have differential prognostic roles in non-small cell lung cancer. *Oncoimmunology*.

[33] Areshkov P. O., Avdieiev S. S., Balynska O. V., Le Roith D., Kavsan V. M. (2012). Two closely related human members of chitinase-like family, CHI3L1 and CHI3L2, activate ERK1/2 in 293 and U373 cells but have the different influence on cell proliferation. *International Journal of Biological Sciences*.

[34] Kang W., Sun T., Tang D., Zhou J., Feng Q. (2019). Time-course transcriptome analysis of gingiva-derived mesenchymal stem cells reveals that Fusobacterium nucleatum triggers oncogene expression in the process of cell differentiation. *Frontiers in cell and developmental biology*.

[35] Fostel L. V., Dluzniewska J., Shimizu Y., Burbach B. J., Peterson E. J. (2006). ADAP is dispensable for NK cell development and function. *International Immunology*.

[36] Ke Z., Wang C., Wu T., Wang W., Yang Y., Dai Y. (2020). PAR2 deficiency enhances myeloid cell-mediated immunosuppression and promotes colitis-associated tumorigenesis. *Cancer Letters*.

[37] Haenisch C., Diekmann H., Klinger M., Gennarini G., Kuwada J. Y., Stuermer C. A. O. (2005). The neuronal growth and regeneration associated Cntn1 (F3/F11/contactin) gene is duplicated in fish: expression during development and retinal axon regeneration. *Molecular and Cellular Neurosciences*.

[38] Liu P., Chen S., Wu W. (2012). Contactin-1 (CNTN-1) overexpression is correlated with advanced clinical stage and lymph node metastasis in oesophageal squamous cell carcinomas. *Japanese Journal of Clinical Oncology*.

[39] Wu H. M., Cao W., Ye D., Ren G. X., Wu Y. N., Guo W. (2012). Contactin 1 (CNTN1) expression associates with regional lymph node metastasis and is a novel predictor of prognosis in patients with oral squamous cell carcinoma. *Molecular Medicine Reports*.

[40] Su J. L., Yang C. Y., Shih J. Y. (2006). Knockdown of contactin-1 expression suppresses invasion and metastasis of lung adenocarcinoma. *Cancer Research*.

[41] Yan J., Wong N., Hung C., Chen W. X. Y., Tang D. (2013). Contactin-1 reduces E-cadherin expression via activating AKT in lung cancer. *PLoS One*.

[42] Su J. L., Yang P. C., Shih J. Y. (2006). The VEGF-C/Flt-4 axis promotes invasion and metastasis of cancer cells. *Cancer Cell*.

[43] Chen D. H., Yu J. W., Wu J. G., Wang S. L., Jiang B. J. (2015). Significances of contactin-1 expression in human gastric cancer and knockdown of contactin-1 expression inhibits invasion and metastasis of MKN45 gastric cancer cells. *Journal of Cancer Research and Clinical Oncology*.

[44] Zhang R., Yao W., Qian P. (2015). Increased sensitivity of human lung adenocarcinoma cells to cisplatin associated with downregulated contactin-1. *Biomedicine & Pharmacotherapy*.

[45] Lankelma J. M., Voorend D. M., Barwari T. (2010). Cathepsin L, target in cancer treatment?. *Life Sciences*.

[46] Sullivan S., Tosetto M., Kevans D. (2009). Localization of nuclear cathepsin L and its association with disease progression and poor outcome in colorectal cancer. *International Journal of Cancer*.

[47] Wang W., Long L., Wang L. (2016). Knockdown of cathepsin L promotes radiosensitivity of glioma stem cells both in vivo and in vitro. *Cancer Letters*.

[48] Ueki N., Wang W., Swenson C., McNaughton C., Sampson N. S., Hayman M. J. (2016). Synthesis and preclinical evaluation of a highly improved anticancer prodrug activated by histone deacetylases and cathepsin L. *Theranostics*.

[49] Sudhan D. R., Pampo C., Rice L., Siemann D. W. (2016). Cathepsin L inactivation leads to multimodal inhibition of prostate cancer cell dissemination in a preclinical bone metastasis model. *International Journal of Cancer*.

[50] Vigano S., Alatzoglou D., Irving M. (2019). Targeting adenosine in cancer immunotherapy to enhance T-cell function. *Frontiers in immunology*.

[51] Martens A., Wistuba-Hamprecht K., Yuan J. (2016). Increases in absolute lymphocytes and circulating CD4+ and CD8+ T cells are associated with positive clinical outcome of melanoma patients treated with ipilimumab. *Clinical Cancer Research*.

[52] Strazzulla A., Barreca G. S., Giancotti A. (2015). Nasopharyngeal carcinoma: review of the literature with a focus on therapeutical implications. *Le Infezioni in Medicina*.

[53] Bergman E. A., Hartana C. A., Johansson M. (2018). Increased CD4(+) T cell lineage commitment determined by CpG methylation correlates with better prognosis in urinary bladder cancer patients. *Clinical Epigenetics*.

[54] Hou Y. C., Chao Y. J., Hsieh M. H., Tung H. L., Wang H. C., Shan Y. S. (2019). Low CD8(+) T cell infiltration and high PD-L1 expression are associated with level of CD44(+)/CD133(+) cancer stem cells and predict an unfavorable prognosis in pancreatic cancer. *Cancers*.

[55] Wang H., Franco F., Ho P. C. (2017). Metabolic regulation of Tregs in cancer: opportunities for immunotherapy. *Trends Cancer*.

[56] Mantovani A., Locati M. (2013). Tumor-associated macrophages as a paradigm of macrophage plasticity, diversity, and polarization. *Arteriosclerosis, Thrombosis, and Vascular Biology*.

[57] Chanmee T., Ontong P., Konno K., Itano N. (2014). Tumor-associated macrophages as major players in the tumor microenvironment. *Cancers (Basel)*.

[58] Sica A., Allavena P., Mantovani A. (2008). Cancer related inflammation: the macrophage connection. *Cancer Letters*.

[59] He B., Di Dong Y. S., Zhou C. (2020). Predicting response to immunotherapy in advanced non-small-cell lung cancer using tumor mutational burden radiomic biomarker. *Journal for immunotherapy of cancer*.

[60] Moik F., Zöchbauer-Müller S., Posch F., Pabinger I., Ay C. (2020). Systemic inflammation and activation of haemostasis predict poor prognosis and response to chemotherapy in patients with advanced lung cancer. *Cancers*.

[61] Perrone F., Minari R., Bersanelli M. (2020). The prognostic role of high blood cholesterol in advanced cancer patients treated with immune checkpoint inhibitors. *Journal for Immunotherapy of Cancer*.

[62] Mildner F., Sopper S., Amann A. (2020). Systematic review: soluble immunological biomarkers in advanced non-small-cell lung cancer (NSCLC). *Critical Reviews in Oncology/Hematology*.

